This article has been retracted.

# TextRank Keyword Extraction Algorithm Using Word Vector Clustering Based on Rough Data-Deduction

**DOI:** 10.1155/2022/5649994

**Published:** 2022-01-25

**Authors:** Ning Zhou, Wenqian Shi, Renyu Liang, Na Zhong

**Affiliations:** School of Electronics and Information Engineering, Lanzhou Jiaotong University, Lanzhou 730070, China

## Abstract

When TextRank algorithm based on graph model constructs graph associative edges, the co-occurrence window rules only consider the relationships between local terms. Using the information in the document itself is limited. In order to solve the above problems, an improved TextRank keyword extraction algorithm based on rough data reasoning combined with word vector clustering, RDD-WRank, was proposed. Firstly, the algorithm uses rough data reasoning to mine the association between candidate keywords, expands the search scope, and makes the results more comprehensive. Then, based on Wikipedia online open knowledge base, word embedding technology is used to integrate Word2Vec into the improved algorithm, and the word vector of TextRank lexical graph nodes is clustered to adjust the voting importance of nodes in the cluster. Compared with the traditional TextRank algorithm and the Word2Vec algorithm combined with TextRank, the experimental results show that the improved algorithm has significantly improved the extraction accuracy, which proves that the idea of using rough data reasoning can effectively improve the performance of the algorithm to extract keywords.

## 1. Introduction

In this information age, people's lives are full of information. Faced with such a huge amount of data, it is particularly important to quickly and accurately obtain the content which we are interested in and which is valuable. As a high-level summary of the text content, keywords can help readers quickly understand the main ideas. In addition, keyword extraction also plays an important role in the fields of information retrieval and text classification. This article mainly discusses the method of using TextRank to extract keywords.

The traditional TextRank algorithm uses the co-occurrence window principle to establish the association between nodes when it is constructing candidate keyword graphs. That is, an edge can be constructed between two nodes in the same window, so the co-occurrence relationship can be used to easily obtain the required graph of word. However, using this principle to judge the correlation between nodes only considers the local relationship, which is relatively limited and may lead to the extraction results being not comprehensive or accurate enough. In addition, the algorithm only uses the information of the document itself. If external knowledge can be introduced into the keyword extraction process of the algorithm, the effect of keyword extraction can be improved in theory.

To solve the above problems and get more accurate extraction results, this paper introduces rough data-deduction theory into the field of text mining for the first time and makes improvements to the TextRank algorithm based on this. Because rough data-deduction has the characteristics of upper approximation and the deduction object is data [1], when the theory is applied to a problem with potential association, it has important application significance for the problem model building and algorithm simulation. However, there are a few application studies on the theory at present, which are only involved in image repair [2] and have not been used in the related research of text language processing. Therefore, it has theoretical and practical significance to improve TextRank algorithm based on rough data-deduction. The algorithm in this paper uses rough data-deduction theory to infer the association relationship between nodes, determine whether there is a potential association between two nodes, and then obtain the transition probability of coverage influences between nodes. At the same time, to make the algorithm consider the influence of external knowledge on keyword extraction, this paper uses the Word2Vec model training to generate word vectors and cluster the word vectors. The TextRank word nodes of graph are nonuniformly weighted according to the clustering distribution of words. Then, we integrate the external world knowledge of a single document into the algorithm and improve the extraction effect of the algorithm. Different from the existing methods that use topic weighting and inverse document frequency weighting to introduce external knowledge, the training data of Word2Vec is independent of the documents to be extracted. Using the word vector generated by it to improve the algorithm, theoretically a more stable extraction result can be obtained.

## 2. Related Work

The Materials and Methods should be described with sufficient details to allow others to replicate and build on the published results. Please note that the publication of your manuscript implicates that you must make all materials, data, computer code, and protocols associated with the publication available to readers. Please disclose at the submission stage any restrictions on the availability of materials or information. New methods and protocols should be described in detail while well-established methods can be briefly described and appropriately cited.

Research manuscripts reporting large datasets that are deposited in a publicly available database should specify where the data have been deposited and provide the relevant accession numbers. If the accession numbers have not yet been obtained at the time of submission, please state that they will be provided during review. They must be provided prior to publication.

The research on keyword extraction methods began at the end of the last century. According to whether it is necessary to provide tagged corpus, keyword extraction can be divided into supervised and unsupervised methods in this paper. The supervised extraction method [3] regards keyword extraction as a binary classification problem to perform binary judgment on the words in the text to determine whether it is a keyword, and this method needs to provide tagged corpus. The unsupervised extraction method does not need to provide tagged corpus. It uses statistical properties to rank the candidate words and takes the most important words as keywords. With the continuous improvement of unsupervised extraction methods, its extraction performance is gradually approaching supervised methods [4], and it has strong adaptability, so it is widely used. This paper focuses on the research of unsupervised extraction algorithms, and the mainstream methods can be summarized into three categories, keyword extraction algorithms based on word frequency statistics [5–8], topic models [9–12], and diagram models [13–17].

There is a big difference between Chinese and English keyword research, and the algorithm based on graph model is a more effective method in the keyword extraction of Chinese text. It can more fully utilize the relationship between text elements than the method based on word frequency statistics, and has a good keyword extraction effect. The TextRank algorithm, as a typical representative based on the word diagram model, has been widely concerned by researchers.

According to the Google's PageRank algorithm, Mihalcea and Tarau proposed the voting algorithm TextRank based on the graph model. In recent years, in order to further improve the keyword extraction effect of the TextRank algorithm, Literature [18] proposed PositionRank, an unsupervised model for extracting keywords from academic documents, which combines information of all locations where words appear to bias PageRank. Literature [19] integrates LDA into the algorithm, taking into account the influence of the subject matter of the whole documentation set, thereby improving the accuracy of extraction. Literature [20] added the time dimension to the algorithm, which can better adapt to changing themes and improve the effectiveness of extraction. Literature [21] introduced word relevance and document language network in the document graph model to improve keyword extraction performance. Literature [22] improved the algorithm based on the theory of basic level category. Literature [23] integrated the location information of the words in the document into the algorithm and improved the effect of the algorithm on keyword extraction. Literature [24] integrated the Doc2Vec model and the K-means algorithm into the algorithm to improve the quality of extraction. In summary, it is found that the improvements of the existing related algorithms are all at the level of combining external features, and fails to start from the inside of the algorithm to improve its accuracy.

With the continuous development of various technologies in the field of artificial intelligence, the neural network tool Word2Vec began to be widely used. Keywords extraction in the text based on the Word2Vec model is one of its important applications. Literature [25] used word2vec to perform K-dimensional vector representation on all the words in the training documentation set, calculated the similarity between words based on the word vectors, and implemented word clustering to get the keywords of the document. Literature [26] combined the LDA topic model with Word2Vec to propose a keyword extraction method that combined topic word embedding and network structure analysis. Literature [27] uses TF-IDF-weighted Glove word vector for word embedding representation. Literature [28] proposed a cuckoo search algorithm and k-means supervised hybrid clustering algorithm to divide all kinds of data samples into clusters so as to provide training subsets with high diversity and merged the word2vec model into the traditional TextRank algorithm by using word embedding technology to improve the accuracy of keyword extraction. Literature [29] merged the word2vec model into the traditional TextRank algorithm by using word embedding technology to improve the accuracy of keyword extraction.

## 3. Research Theory

### 3.1. TextRank Algorithm

The TextRank [30] algorithm is a graph model sorting algorithm based on the Google PageRank [31, 32] algorithm. Now it is widely used in the field of keyword extraction [33, 34]. The basic idea of the algorithm is the voting principle. First, the target text is divided into several meaningful words, and the local connection between the words, which is the same as co-occurrence window, is used to determine the association between the candidate words and construct the candidate word graph. Then, our algorithm uses the voting mechanism to sort the candidate words to achieve keyword extraction. The main steps are as follows:

(1) Sentence segmentation: Segment the target text *T* according to the completeness of the sentence, that is, *T*=[*S*_1_, *S*_2_,…, *S*_*m*_].
(2) Word segmentation and filtering: Segment word for each sentence, *S*_*i*_ ∈ *T*, and tag part-of-speech, then filter out stop words and some words that are not included in the specified part-of-speech, that is, *S*_*i*_=[*t*_*i*,1_, *t*_*i*,2_,…, *t*_*i*,*n*_], where *t*_*i*,*j*_ is the candidate keyword after filtering.
(3) Construct graph: Construct candidate graph of word, *G* = (*V*, *E*), where *V* is the vertex set which is composed of the candidate words obtained in (2), *E* is the edge set which is a subset of *V* × *V*. The traditional algorithm uses the co-occurrence window to construct the edges between two nodes in the graph. That is, only when the candidate words corresponding to the two nodes appear in a window whose length is *K*, there is an edge between the two nodes, where *K* is the window size and determines the maximum number of words that can co-occur.
(4) Iterative calculation: Iteratively calculate the weight of each node according to formula (1) [30] until the calculation result converges.
  (1) $$\begin{array}{c} WS\left(v_{i}\right)=\left(1-d\right)+d\times \underset{v_{j}\in In\left(v_{i}\right)}{\sum }\frac{w_{ji}}{\sum_{v_{k}\in \text{Out}\left(v_{i}\right)}w_{jk}}WS\left(v_{i}\right). \end{array}$$
In the formula, In(*v*_*i*_) represents the node set pointing to node *v*_*i*_, and *d* ∈ [0,1] is the damping factor, which was originally the random walk probability of the PageRank algorithm. The original intention of the setting is to prevent those pages without external links from swallowing the opportunity for users to browse down. There are also nodes without any pointing in the text graph model, the general value is 0.85. If there is a node in the candidate word graph whose error rate is less than a specific limit value, it is considered that the node has reached convergence, and this limit value is usually set to 0.0001. *p*(*v*_*j*_⟶*v*_*i*_) represents the jump probability from node *v*_*j*_ to *v*_*i*_, which is calculated by formula (2) in the traditional TextRank algorithm.
  (2) $$\begin{array}{c} p\left(v_{j}⟶v_{i}\right)=\left\{\begin{array}{cc} \frac{w_{ji}}{\sum_{v_{k}\in \text{Out}\left(v_{j}\right)}w_{jk}}, & \;if\;\exists \left(v_{j}⟶v_{i}\right)\in E\\ 0, & \text{otherwise} \end{array}\right\}. \end{array}$$
In the formula, Out(*v*_*j*_) represents the set of nodes which is pointed by *v*_*j*_, *w*_*ji*_ represents the weight of the edge from node *w*_*j*_ to node *w*_*i*_, which is determined by the co-occurrence of two words in the traditional algorithm.
(5) Sorting: Sort the node weights in reverse order and use the first K word as keyword in the target text.

### 3.2. Rough Data-Deduction

#### 3.2.1. Rough Set Theory

The original application of rough set theory in text processing is to classify texts to speed up the classification and improve the accuracy of classification [35]. The idea of rough data-deduction is based on rough set theory, and integrates the approximate information in the upper approximation concept into the process of data reasoning. Therefore, the introduction of concepts related to rough set theory will play a role in understanding rough data-deduction. Here is a brief introduction to some related knowledge in the rough set.

Let *U* be a dataset and *R* an equivalence relation on *U*. The structure composed of *U* and *R* is called approximation space denoted by *M*=(*U*, *R*), and *U* is the domain of discourse. Let *U*/*R*={[*a*]_*R*_*|a* ∈ *U*} be referred to as the partition of *U* relative to *R*, where [*a*]_*R*_ is the *R*-equivalence class and determined by *a*. For any subset *X*⊆*U* of *U*, in approximate space *M*, the upper and lower approximation *R*_*∗*_(*x*) of *X* are defined in the following ways [36]:

(3) $$\begin{array}{c} R^{*}\left(x\right)=\cup^{}\left\{\frac{{\left[a\right]}_{R}|{\left[a\right]}_{R}\in U}{R\text{ and }{\left[a\right]}_{R}\cap^{}X\neq \phi }\right\},\\ R_{*}\left(x\right)=\cup^{}\left\{\frac{{\left[a\right]}_{R}|{\left[a\right]}_{R}\in U}{R\text{ and }{\left[a\right]}_{R}\subseteq^{}X\neq \phi }\right\}. \end{array}$$

That is, the upper approximation of the subset *X* is equal to the union of all R-equivalence classes whose intersection with *X* is not equal to the empty set, and the lower approximation of the subset *X* is equal to the union of all R-equivalence classes contained in *X*.

The lower approximation *R*_*∗*_(*x*) is approaching *X* from the inside of *X*, and the upper approximation *R*^*∗*^(*x*) is approaching from the outside of *X*. If *X* is considered to contain precise information, *R*_*∗*_(*x*) contained within *X* is often more accurate than precise information. *R*^*∗*^(*x*) expands the scope of precise information to include external information, so that the concept of rough set can be derived. That is, when *R*^*∗*^(*x*) ≠ *R*_*∗*_(*x*), *X* is called a rough set. And, when *R*^*∗*^(*x*)=*R*_*∗*_(*x*), *X* is called a definite set [36]. Since the information of *R*_*∗*_(*x*) is too accurate, the information in *R*^*∗*^(*x*) covers *X* which is an extension of accurate information. Therefore, incorporating *R*^*∗*^(*x*) into rough data-deduction can increase the deduction data and expand the deduction range, and the results obtained will be more accurate.

#### 3.2.2. Rough Deduction-Space

Rough deduction-space is the structure space that rough data-deduction depends on, and it is an expansion of an approximation space *M*=(*U*, *R*) in content and structure. Then, in the formula, *K*={*R*_1_, *R*_2_,…, *R*_*n*_}(*n* ≥ 1), where *R*_*i*_(*i*=1,2,…, *n*) is an equivalence relation on *U*. Given a binary relation *S*⊆*U* × *U*, *S* is referred to as a deduction relation. The structure composed of *U*, *K*, and *S* is called a rough deduction-space denoted by *W*=(*U*, *K*, *S*) [1].

### 3.3. Rough Data-Deduction

Rough data-deduction accomplishes deductions from data to data, which is different from any logical deduction in the mathematical logic. Since most things and objects in real life can be abstracted as data, data-oriented reasoning is more widely used. Let *W*=(*U*, *K*, *S*) be rough deduction-spaces, *a* ∈ *U* and *R* ∈ *K*, then rough data-deductions are defined as follows:

1. Let *b* ∈ *U*, if *b* ∈ *R*^*∗*^([*a* − *R*]), *a* can directly get rough deduction *b* with respect to *R*, denoted by *a*⇒_*R*_*b*, where [*a* − *R*]={*x|x* ∈ *U*,  and there is a data *z* ∈ [*a*]_*R*_ making *z*, *x* ∈ *S*}.The subset [*a* − *R*] is called the S-predecessor set of [*a*]_*R*_.
2. Let *b*_1_, *b*_2_, ..., *b*_*n*_, *b* ∈ *U*, if *a*⇒_*R*_*b*_1_, *b*_1_⇒_*R*_*b*_2_,…, and *b*_*n*−1_⇒_*R*_*b*_*n*_*b*_*n*_⇒_*R*_*b*(*n* ≥ 0),  a roughly deduces *b* with respect to *R*, which is denoted by *a|*=_*R*_*b*.
3. For *R* ∈ *K* and *a*, *b* ∈ *U*, the process of deduction whether *a* roughly deduces *b* with respect to (1) or (2) is called the rough data-deduction with respect to *R* in *W*=(*U*, *K*, *S*), or rough data-deduction for short [1].

Rough data-deduction can expand association scope and increase association data. If this theory is applied to the TextRank keyword extraction algorithm, the association between nodes of two words can be obtained through deduction from the overall situation. According to this, the graph of candidate keywords is constructed to extract keywords, and the extraction result should be more comprehensive.

### 3.4. Word2Vec

Word2Vec is a model tool for word vector training open sourced by Google. It can vectorize all words to quantitatively measure the relationship between words and explore the relationship between candidate words. It uses a shallow neural network model to automatically learn the occurrence of words in the corpus, and embeds the words into a space with a moderate dimension, that is, words⟶*R*^*n*^, and the expression result of the words in the new space *R*^*n*^ is the word vector [37].

The idea of Word2Vec [26, 36] comes from the probability calculation of Bayesian occurrence estimation, let *T*=*w*_1_, *w*_2_,…, *w*_*n*_ be sentences including *n* words, the probability of occurrence of the sentence *T* is:

(4) $$\begin{array}{c} P\left(T\right)=\overset{n}{\underset{i=1}{\prod }}p\left(w_{i}|w_{i-n-1}w_{i-n-2},\ldots ,w_{i-1}\right). \end{array}$$

And, the Bayesian estimation of the occurrence chance of *w*_*i*_ is

(5) $$\begin{array}{c} p\left(w_{i}|w_{i-n-1}w_{i-n-2},\ldots ,w_{i-1}\right)=\frac{C\left(w_{1}w_{2},\ldots ,w_{n}\right)}{C\left(w_{1}w_{2},\ldots ,w_{n-1}\right)}. \end{array}$$

In the formula, *C*(*w*_1_*w*_2_,…, *w*_*n*_) is the probability of the sentence *w*_1_*w*_2_,…, *w*_*n*_ in the corpus.

The Word2Vec tool mainly includes the following two training modes: Continuous Bag-of-Words (CBOW) and Skip-Gram, both of which are three-layer neural networks (input layer, projection layer, and output layer). The CBOW model [25, 36] predicts the current value through context, that is, inputting a known context and outputting the prediction of the current word, as shown in Figure 1. What is predicted by the CBOW model in the figure is *p*(*w*_*t*_*|w*_*t*−2_, *w*_*t*−1_, *w*_*t*+1_, *w*_*t*+2_), and the window is 2. Assuming that *k* words are taken before and after the target word *w*_*t*_, that is, the window size is *k*, the prediction of the CBOW model is

(6) $$\begin{array}{c} p\left(w_{t}|w_{t-k},w_{t-\left(k-1\right)},\ldots ,w_{t-1},w_{t+1},\ldots ,w_{t+\left(k-1\right)},w_{t+k}\right). \end{array}$$

And, the learning goal of this model is to maximize the function *L*_1_:

(7) $$\begin{array}{c} \;L_{1}=\overset{V}{\underset{t=1}{\prod }}p\left(w_{t}|w_{t-k},w_{t-\left(k-1\right)},\ldots ,w_{t-1},w_{t+1},\ldots ,w_{t+\left(k-1\right)},w_{t+k}\right). \end{array}$$

The Skip-Gram model [25, 36] has the opposite characteristics of the CBOW model. Its input is a word vector of a specific word, and the output is a context word vector corresponding to a specific word, as shown in Figure 1. Similarly, if it is assumed that *k* words are taken before and after the word *w*_*t*_, that is, the window size is *k*, then the prediction of the Skip-Gram model is

(8) $$\begin{array}{c} p\left(w_{t+p}|w_{t}\right)\left(-k\leq p\leq k,k\neq 0\right). \end{array}$$

And, the learning goal of this model is to maximize the function *L*_2_:

(9) $$\begin{array}{c} L_{2}=\overset{V}{\underset{t=1}{\prod }}\overset{k}{\underset{p=-k,t\neq 0}{\prod }}p\left(w_{t+p}|w_{t}\right). \end{array}$$

CBOW and Skip-Gram are two important models in Word2Vec, which describe the association between surrounding words and current words from different angles. Comparing the two models, the Skip-Gram model can generate more training samples and capture more semantic details between words. Under ideal conditions where the corpus is good enough, the Skip-Gram model is superior to the CBOW model. However, in the case of less corpus, it is difficult to capture more details between words. On the contrary, the CBOW model has the characteristics of averaging which will make the training effect better, and this study considers both. At the same time, two optimization methods are proposed to reduce the training complexity: negative sampling [38] and hierarchical softmax [39] to speed up the training process.

Compared with the traditional text representation, Word2Vec generates a word vector with a lower dimension, and the semantic and syntactic relationship between words can also be well reflected in the vector space, because the words with similar semantics are close to each other in space. It can be said that the word vectors learned in Word2Vec training contain the semantic information of the words in the dataset. Pretraining language models such as GPT and BERT have better training effects, but their data scale is large. Therefore, this paper weights the jump probability between TextRank word graph nodes based on the relationship between the text word vectors obtained by Word2Vec training.

## 4. Improved Algorithm Using Word Vector Based on Rough Data-Deduction

The classic TextRank algorithm constructs the graph model of candidate keywords through the co-occurrence relationship and then iteratively calculates the weight of each node through the average transition probability matrix until it converges. This approach is relatively simple and effective, but it has certain limitations. The rule of co-occurrence window only considers the correlation between local words, so some words that are locally associated with certain keywords may be extracted. However, the keywords of a document are not limited to some words around important words. When extracting text keywords, we must fully consider the words in the text and some potentially associated words. Words with potential association will have an important impact on the entirely iterative sorting process, and this potential association can be explored through the theory of rough data-deduction. At the same time, considering the influence of external knowledge on keyword extraction, the improved algorithm introduces Word2Vec to quantify the candidate word nodes. Unlike existing methods that use topic weighting and inverse document frequency weighting to introduce external knowledge, the training data of the Word2Vec model is independent of the text data to be extracted. Using the word vectors generated by its training to improve the algorithm, in theory, a more stable extraction result can be obtained [40]. The word vector reflects the external knowledge information, and the candidate keywords can be clustered into several clusters according to the similarity between the word vectors. The farther a word is from the centroid of the cluster, the more it can reflect the different aspects of a cluster from words near the centroid. When it is used as a word node in TextRank, the higher the importance of its vote, the higher the probability of jumping between adjacent nodes.

First, starting from the meaning of the words, according to the similarity of the meanings between words, the candidate keywords are classified. Since a group of different words with similar meanings may describe the same important content in a document, the weight of this group of words should be increased accordingly to improve the accuracy of the extraction results. The classic TextRank algorithm does not consider this aspect but only considers the word itself, thereby ignoring the contribution rate of words with similar meanings. The improved algorithm takes the word meaning into account and divides the candidate words by word meaning to participate in the subsequent association deduction, which can extract keywords more effectively.

Second, the rough deduction-space *W*=(*U*, *K*, *S*) is introduced to describe the structure of keyword extraction, where *U* is a dataset composed of candidate keywords, *K* is the set of equivalence relations, and *R* ∈ *K*, for *a*, *b* ∈ *U*, 〈*a*, *b*〉 ∈ *R* if and only if *a* and *bb* have similar meanings. *S*⊆*U* × *U* is defined as *S*={〈*u*, *v*〉*|u*, *v* ∈ *U* and there is an association between *u* and *v*}.

At the same time, using rough data-deduction, it is assumed that the deduction relationship is

(10) $$\begin{array}{c} S=\left\{\langle w_{1},w_{4}\rangle ,\langle w_{3},w_{4}\rangle ,\langle w_{3},w_{6}\rangle ,\langle w_{5},w_{8}\rangle \right\}, \end{array}$$

where *w*_1_ ~ *w*_9_ are candidate keywords selected from the text after word segmentation and filtering, and this deduction relationship is determined by the association degree of the association rules in the deduction, that is, point mutual information. For the equivalence relation *R* ∈ *K*, it is assumed that the division of U with respect to *R* is

(11) $$\begin{array}{c} \frac{U}{R}=\left\{\left\{w_{1},w_{2},w_{3}\right\},\left\{w_{4},w_{5},w_{6}\right\},\left\{w_{7},w_{8},w_{9}\right\}\right\}. \end{array}$$

The equivalence division here is based on the similarity of word meanings between candidate words, combined with the above information to obtain a rough data-deduction schematic diagram in keyword extraction, as shown in Figure 2.

As shown in Figure 2, in the process of rough data-deduction, for the candidate word *w*_1_, the algorithm obtains *w*_2_, *w*_3_ based on the similarity rule of word meaning, so *w*_1_, *w*_2_, and *w*_3_ are divided into a dataset. Similarly, *w*_4_ ~ *w*_9_ can be divided. Based on the association degree of association rules in point mutual information deduction, the algorithm deduces from *w*_1_ to *w*_4_ and get *w*_5_ ~ *w*_9_. According to the definition of rough data-deduction, for *w*_1_, there are [*w*_1_]_*R*_={*w*_1_, *w*_2_, *w*_3_}, [*w*_1_ − *R*]={*w*_4_, *w*_6_}, *R*^*∗*^([*w*_1_ − *R*])={*w*_4_, *w*_5_, *w*_6_}, so *w*_1_⇒_*R*_*w*_5_. For candidate word *w*_5_: [*w*_6_]_*R*_={*w*_4_, *w*_5_, *w*_6_}, [*w*_5_ − *R*]={*w*_8_}, *R*^*∗*^([*w*_5_ − *R*])={*w*_7_, *w*_8_, *w*_9_}, so *w*_5_⇒_*R*_*w*_9_. Finally, *w*_1_*|*=_*R*_*w*_9_ can be got from *w*_1_⇒_*R*_*w*_5_ and *w*_5_⇒_*R*_*w*_9_. As can be seen from the above, there is also a potential correlation between *w*_1_ and *w*_9_, which can provide a certain contribution for the calculation. The association between candidate keywords is established by the above rules, and the association weight can be added as a contribution rate to the iterative calculation process to improve the accuracy of extraction. For any two nodes *v*_*j*_ and *v*_*i*_, the influence of node *v*_*j*_ on *v*_*i*_ is transmitted through its directed edge 〈*v*_*j*_, *v*_*i*_〉, and the weight of the edge determines the influence of *v*_*j*_ and finally obtained by *v*_*i*_. Therefore, let the association weight between *v*_*j*_ and *v*_*i*_ based on rough data-deduction be the weight of the coverage influence of node *v*_*j*_ transmitted to node *v*_*i*_, and record it as *w*_*ij*_′. With reference to formula (2), the transition probability of coverage that influences between candidate keywords nodes *v*_*j*_ and *v*_*i*_ is

(12) $$\begin{array}{c} p_{\mathrm{cov}}\left(v_{j}⟶v_{i}\right)=\frac{w_{jk}^{\prime }}{\sum_{v_{k}\in \text{Out}\left(v_{j}\right)}w_{jk}^{\prime }}. \end{array}$$

Then, for the text *T* and its candidate keyword word set {*w*_1_, *w*_2_,…, *w*_*n*_} and the Word2Vec word vector model obtained by training, let $\overset{⟶}{w_{i}}$ represent the word vector corresponding to the word *w*_*i*_, {*C*_1_, *C*_2_,…, *C*_*k*_} represent the clustering result after K-means clustering by the word vector set of the text, and formula (13) is proposed to calculate the voting importance of any word *v*_*i*_ in the cluster *C*_*v*_*i*__.

(13) $$\begin{array}{c} c\text{ weight}\left(v_{i}\right)=\frac{d\left(\overset{⟶}{v_{i}},\overset{⟶}{c_{v_{i}}}\right)}{\sum_{v_{j}\in c_{v_{i}}}d\left(\overset{⟶}{v_{i}},\overset{⟶}{c_{v_{i}}}\right)}\times \left|C_{v_{i}}\right|. \end{array}$$

In this formula, $\overset{⟶}{C_{v_{i}}}$ is the vector corresponding to the centroid of cluster *C*_*v*_*i*__, $d\left(\overset{⟶}{v_{i}},\overset{⟶}{c_{v_{i}}}\right)$ is the Euclidean distance from vector $\overset{⟶}{v_{i}}$ to vector $\overset{⟶}{c_{v_{i}}}$ in the word vector space, and |*C*_*v*_*i*__| is the number of words included in the cluster *C*_*v*_*i*__. The total voting score of a cluster is the number of nodes in the cluster, and the voting weight of each node in the cluster is proportionally distributed according to the Euclidean distance from the centroid. The further away from the centroid, the higher the importance of voting. When the semantic association of the two nodes in the word vector space is expressed as the clustering weighted influence between the nodes, then through cluster analysis and calculation to get the voting importance of each word, the transition probability of cluster influence between nodes *v*_*j*_ and *v*_*i*_ is

(14) $$\begin{array}{c} p_{\text{clu}}\left(v_{j}⟶v_{i}\right)=\frac{c\text{ weight}\left(v_{i}\right)}{\sum_{v_{k}\in \text{out}\left(v_{j}\right)}c\text{ weight}\left(v_{k}\right)}. \end{array}$$

Finally, according to the coverage influence between nodes and clustering weighted influence, formula (15) is proposed to calculate the jump probability between nodes *v*_*i*_ and *v*_*j*_.

(15) $$\begin{array}{c} p\left(v_{j}⟶v_{ji}\right)=\alpha \times p_{\mathrm{cov}}\left(v_{j}⟶v_{i}\right)+\beta \times p_{\text{clu}}\left(v_{j}⟶v_{i}\right). \end{array}$$

In this formula, *α* and *β* are the weight coefficients of each influence, respectively, and *α*+*β*=1. This paper takes *α*=0.7 and *β*=0.3 according to the result of experiments.

According to the theory of link analysis, as long as the jump probability transition matrix between nodes in a given graph is given, the importance of the nodes can be calculated iteratively by formula (1).

The main steps to improve the algorithm are as follows:

**Step 1 .**

Preprocess the target text based on the classic TextRank algorithm, to get candidate keywords by cutting sentences, word segmentation, and part-of-speech filtering.

**Step 2 .**

Divide the candidate keywords into different equivalence classes according to the similarity of word meanings. In this paper, we divide words based on HowNet and Cilin. For any two words *w*_1_, *w*_2_, the division rule [41] is

(16) $$\begin{array}{c} s=\lambda_{1}s_{1}+\lambda_{2}s_{2}. \end{array}$$

In this formula, *s*_1_ and *s*_2_ are the similarity calculated by HowNet and Cilin, respectively, *λ*_1_ and *λ*_2_ are the two weights given to *s*_1_ and *s*_2_, and the requirement *λ*_1_+*λ*_2_=1. The values of *λ*_1_ and *λ*_2_ are defined by the distribution of words *w*_1_ and *w*_2_ in HowNet and Cilin in Figure 3.

In this formula, the strategies for taking the value of *λ*_1_ and *λ*_2_ are as follows [41]:

1. When *w*_1_ ∈ *C*, *w*_2_ ∈ *C*, calculate the similarity between *w*_1_ and *w*_2_, respectively, based on HowNet and Cilin. Then, denote them as *s*_1_ and *s*_2_. Takes *λ*_1_=*λ*_2_=0.5 in the experiment of this paper.
2. When *w*_1_ ∈ *A*, *w*_2_ ∈ *A* or *w*_1_ ∈ *B*, *w*_2_ ∈ *B*, calculate the similarity between *w*_1_ and *w*_2_ based on HowNet or Cilin, and denote them as *s*_1_ or *s*_2_. Here, *λ*_1_ is 1 and *λ*_2_ is 0.
3. When *w*_1_ ∈ *A*, *w*_2_ ∈ *B*, find the synonyms set of *w*_2_ based on Cilin, then calculate the similarity of these synonymous words with *w*_1_ based on HowNet, and take the maximum value as *s*_1_. If *w*_2_ has no synonymous words in Cilin, then take *s*_1_=0.2. Now *λ*_1_=1 and *λ*_2_=0.
4. When *w*_1_ ∈ *A*, *w*_2_ ∈ *C*, first calculate the similarity between *w*_1_ and *w*_2_ based on HowNet and denote as *s*_1_. Then, find the synonyms set of *w*_2_ in Cilin and calculate the similarity with *w*_1_ based on HowNet. Take the maximum value and denote as *s*_2_. If *w*_2_ has no synonymous words in Cilin, then take *s*_2_=*s*_1_. Now *λ*_1_ > *λ*_2_. Takes *λ*_1_=0.6 and *λ*_2_=0.4 in the experiment of this paper.
5. When *w*_1_ ∈ *B*, *w*_2_ ∈ *C*, first calculate the similarity between *w*_1_ and *w*_2_ based on Cilin and denote as *s*_2_. Then, find the synonyms set of *w*_1_ in Cilin and calculate the similarity with *w*_2_ based on HowNet. Take the maximum value and denote as *s*_1_. If *w*_1_ has no synonymous words in Cilin, then take *s*_1_=*s*_2_. Now *λ*_2_ > *λ*_1_. Takes *λ*_1_=0.4 and *λ*_2_=0.6 in the experiment of this paper.

The calculation of word similarity based on HowNet is as follows [41]:

(17) $$\begin{array}{c} \text{sim}\left(C_{1},C_{2}\right)=\sum_{i=1}^{3}\beta_{i}\prod_{j=1}^{i}{\text{sim}}_{j}\left(C_{1},C_{2}\right). \end{array}$$

(18) $$\begin{array}{c} \text{sim}\left(W_{1},W_{2}\right)=\underset{i=1,\ldots ,m,j=1,\ldots ,n}{\max}\left\{\text{sim}\left(C_{1i},C_{2j}\right)\right\}. \end{array}$$

In formula (17), sim_1_(*C*_1_, *C*_2_) is the similarity calculated by the set of independent sememe, sim_2_(*C*_1_, *C*_2_) is the similarity of the characteristic structure of the relational sememe, and sim_3_(*C*_1_, *C*_2_) is the similarity of the characteristic structure of the relation symbol. The parameter *β*_*i*_(1 ≤ *i* ≤ 3) is adjustable and satisfies *β*_1_+*β*_2_+*β*_3_=1. After experiments, *β*_1_, *β*_2_, and *β*_3_ in the algorithm of this paper take 0.7, 0.17, and 0.13, respectively. Formula (17) obtains the similarity of sense. When there are multiple senses in a word, formula (18) is used to calculate the maximum similarity value among all sense combinations, which is the similarity of two words, where *m* is the number of senses of the word *W*_1_ and *n* is the number of senses of the word *W*_2_

The calculation of word similarity based on Cilin is as follows [40]:

(19) $$\begin{array}{c} \text{sim}\left(C_{1},C_{2}\right)=\left(1.05-0.05\text{ dis}\left(C_{1},C_{2}\right)\right)\sqrt{e^{-k/2n}}. \end{array}$$

In formula (19), dis(*C*_1_, *C*_2_) is the distance function of word coding *C*_1_ and *C*_2_ in the tree structure; *n* is the total number of nodes in the branch layer, which indicates the number of direct children of the nearest common parent node adjacent between two words; *k* represents the separation distance between the branches where the two words are located in the nearest common parent node. Similarly, when a word corresponds to multiple codes, formula (18) is used to calculate the similarity of words.

**Step 3 .**

The association degree of the association rules in rough reasoning is defined as [42]

(20) $$\begin{array}{c} \text{PMI}\left(A,B\right)=\frac{p\left(A,B\right)}{p\left(A\right)p\left(B\right)}. \end{array}$$

In this formula,  *A*  and *B* are two candidate keywords in the text, *p*(*A*, *B*) represents the frequency of occurrence of *A* and *B* in the same sentence, *p*(*A*) is the frequency of occurrence of *A* and *p*(*B*) is the frequency of occurrence of *B*. The larger the PMI value, the more relevant.

According to this degree of association, it is determined that there are candidate keywords that are directly related. That is, when PMI(*w*_1_, *w*_2_) ≠ 0, there is a direct association between *w*_1_ and *w*_2_, then *w*_1_, *w*_2_ and their association weight *w*_*ij*_′ are stored into the association set. At the same time, the deduction relationship *S* for rough data-deduction can be established according to this association weight. Next, the rules of rough data-deduction are used to obtain the association between the remaining candidate keywords in all different equivalence classes, and these words and their association weight *w*_*ij*_′ are also stored in the association set. The transition probability of coverage influence between candidate keyword nodes is obtained by formula (12).

**Step 4 .**

The popular Python software package Gensim is used to train and construct the Word2vec model, and the largest Wikipedia online open knowledge base is selected as the training corpus, which can ensure that the model has better generalization ability. The Word2Vec model is trained to generate word vectors, then the *K*-means clustering is performed on the word vectors of the candidate words, and the transition probability of clustering influence between the candidate keyword nodes is obtained from formulas (14) and (15).

**Step 5 .**

The jump probability between word nodes is obtained by formula (16). Finally, the weight of each candidate keyword is iteratively iterated to convergence using formula (1). The flow chart of the improved algorithm is shown in Figure 4.

## 5. Experimental Results and Analysis

### 5.1. Experimental Data and Evaluation Criteria

#### 5.1.1. Experimental Data

The experiment selected the Wikipedia Chinese corpus released in February 2020 “zhwiki-20200201-pages-articles-multistream.xml.bz2” to train Chinese word vectors [43, 44], which contains a main file of 1.9CB. First, the experiment uses the Python software package Gensim to convert the downloaded xml compressed file to txt format. Second, it uses opencc to simplify the wiki content and remove other characters except Chinese characters. Finally, after using the jieba word segmentation tool [45] to segment the Chinese corpus obtained above, the word vector is trained using the Word2Vec tool [46]. And, the following datasets were used in the experiment to test the extraction results of each algorithm.

Dataset 1: The experiment selected 1.4 GB of SogouCA from Sogou Lab as the basis for extracting the test text. The dataset contains news data on various fields from June to July 2012, related to domestic and foreign agencies, sports, culture, entertainment, etc. A total of 2045 texts in various fields were randomly selected to form a test set to test the effect of the algorithm. At the same time, many teachers and students with undergraduate degree or above are invited. They are all teachers and students of the Department of Journalism and Chinese of our school. Using manual cross-labeling, 10 keywords are extracted for each text and given in order of importance.

In addition, in order to prevent overfitting of the experimental results of the improved algorithm, the experiment also tested the extraction effect of the improved algorithm based on the following two different types of datasets:

Dataset 2: In this paper, we use CNKI as the retrieval platform and use advanced search method to randomly collect the text data needed by the experiment in the following types of literature, namely, “Geology,” “General Chemistry Industry,” “Highway and Waterway Transportation,” “Fundamental Science of Agriculture,” “Plant Protection,” “Paediatrics,” “Cardiovascular System Disease,” “Geography,” “Biography,” “Military Affairs,” “Chinese Communist Party,” “Ideological & Political Education,” “Computer Hardware Technology,” “Internet Technology” and “Market Research and Information.” From the result set, we selected the titles, abstracts, and keywords of the journal texts in the period from 2014 to 2020 and graded in CSCD/CSSCI and above. And, we exclude texts whose abstract length is less than 150 words and documents whose number of manually marked keywords is less than or equal to 1. The final test dataset contains 17514 data and 65310 keywords provided by the author, and each paper contains 3.73 keywords.

Dataset 3: The Python web crawler is used to capture user comment data of some restaurants in the Taiyuan area of Dianping, including 400 restaurants and 120,000 user comments. However, some of the restaurants only have a very small number of user reviews, which will affect subsequent experiments, so they are excluded from the dataset. In addition, since many users only score the merchants without writing specific review content, user reviews are empty. These kinds of data are also not conducive to subsequent experiments, so it is cleaned from the dataset. The final test dataset contains 17,309 valid user reviews of 178 merchants. At the same time, teachers and students who have manually labeled keywords for dataset 1 are asked to label valid keywords for this dataset [47].

#### 5.1.2. Evaluation Criteria

In addition, the article uses three evaluation indicators commonly used in the field of information retrieval and classification to compare the quality of the experimental results. It contains the precision (*P*), which represents the accuracy of the extraction results; the recall (*R*), which represents the degree of coverage of the extraction results for the correct keywords; and the *F*-Measure (*F*), which is a comprehensive evaluation index of the reconciliation of *P* and *R*. The specific calculation formulas of the three indicators are as follows [48–50]:

(21) $$\begin{array}{c} P=\frac{K_{A}\cap^{}\;K_{B}}{K_{B}}\times 100\%,\\ R=\frac{K_{A}\cap^{}\;K_{B}}{K_{A}}\times 100\%,\\ F=\frac{2\times P\times R}{P+R}\times 100\%. \end{array}$$

In this formula, *K*_*A*_ represents the set of manually annotated keywords, and *K*_*B*_ represents the set of keywords extracted by the algorithm.

The operating system of the experimental environment is Windows7-64bit. The algorithm proposed in this paper is implemented in Python language. The word segmentation and part-of-speech tagging use Jieba open source tools. At the same time, the remaining contrast algorithms involved in the experiment are completed using python language.

### 5.2. Experimental Results and Analysis

#### 5.2.1. Determine the Weight Coefficient *α*, *α*, *β*. *β*

In this paper, the transition probability of coverage influence obtained by rough data-deduction and the transition probability of cluster influence obtained by word vector clustering are used to jointly determine the jump probability between nodes. The value of the jump probability directly affects the extraction effect of the improved algorithm, so it is very important to determine the value of the weight coefficient in formula (15). Based on dataset 1, the number of extracted keywords is set to 3–10, and the following 11 groups of *α* and *β* values are tested: *E*_1_ (1.0, 0), *E*_2_ (0.9, 0.1), *E*_3_ (0.8, 0), *E*_4_ (0.7, 0.3), *E*_5_ (0.6, 0.4), *E*_6_ (0.5, 0.5), *E*_7_ (0.4, 0.6), *E*_8_ (0.3, 0.7), *E*_9_ (0.2, 0.8), *E*_10_ (0.1, 0.9), and *E*_11_ (0, 1.0). The *F*-Measure of the extraction result of the improved algorithm corresponding to each set of data is shown in Figure 5.

It can be seen from Figure 5 that the extraction effect of the algorithm in this paper is different under different values of *α* and *β*. In the experiment, the weighting coefficients are compared under the same test set. And, it is found that when the fifth set of data *E*_4_ (0.7, 0.3) is taken, the algorithm of this paper has the best extraction effect. Therefore, the algorithm takes *α*=0.7 and *β*=0.3 in this paper.

#### 5.2.2. Comparative Algorithm

Based on the same test set, this paper compares the following algorithms with the experimental results of this algorithm.

## 6. Experimental Results

The value of two important parameters in the experiment will affect the extraction result of the TextRank algorithm, which includes the co-occurrence window size *ω* and the number of keywords *k*. However, the implementation of the TF-IDF algorithm based on statistical characteristics and the algorithm in this paper are not affected by the parameter *ω*. For the determination of the parameter *ω*, we set the number of extracted keywords as *k* = 10 based on dataset 1, and when the window value is within [6, 12], we compare the *F*-Measure of the extraction result of the algorithm. The comparison results are shown in Figure 6.

It can be seen from Figure 6 that the extraction effect of the TextRank algorithm is different under different values of *ω*. This paper compares the extraction effects of different values of *ω* under the same test set, and finds that the TextRank algorithm has the best extraction effect when *ω*=6. Therefore, in order to ensure the effectiveness of the algorithm in this paper, the initial value of *ω* of the TextRank algorithm in the comparative experiment is set to 6. At the same time, the other parameters involved in the contrast algorithm are taken from the optimal values used in the respective literature. When the number of keywords is within [3.10], we calculate the precision (*P*), recall (*R*), and *F*-Measure (*F*) of the following nine algorithms. The experimental results (retain two decimal places) are shown in Table 1.

At the same time, in order to comprehensively observe the differences of different keyword extraction methods, the author further gives the overall changes of the *P*, *R* , and *F*-Measure of nine methods when the top *N* value is [3, 10] in the form of line chart, as shown in Figures 7–9.

Figure 7 describes the changing trend of the accuracy of each algorithm when extracting different numbers of keywords. It can be seen from the figure that as the number of extracted keywords increases, the accuracy of each algorithm decreases to some extent. However, the accuracy of the RDD-WRank algorithm in this paper is higher than that of the other algorithms. Because the rough data-deduction rules adopted by the algorithm in this paper will incorporate the approximate information into the process of data deduction, it can make the mutual inference between the data show the characteristics of approximate implication or imprecise association, and explore potential association between candidate keywords. If the potential association is added to the iterative calculation of the weight of each candidate keyword, a more accurate extraction result will be obtained. Therefore, the accuracy of the algorithm in this paper will be higher in theory than the algorithms that calculate the association between words according to fixed association rules or rely on statistical word frequency, and its *P* value will be higher than that of the other algorithms.

Figure 8 describes the changes in the recall of each algorithm when extracting different numbers of keywords. The recall of the RDD-Wrank algorithm in this paper is higher than that of the other several algorithms. At the same time, as the number of keywords increases, the relative increase of the algorithm's recall rate becomes more obvious. This is because the TF-IDF algorithm is too dependent on the word frequency and does not consider the association between words at all. Although the improved algorithms that retain the principle of the co-occurrence window of the traditional TextRank algorithm consider the relationship between words, the algorithm is more inclined to propose frequent words because of the limitations of the association rules adopted by the algorithm. This may ignore important words that have a low frequency but can describe the subject of the text. The rough data-deduction used in the RDD-WRank algorithm can expand the scope of association and increase the association data, which can enhance the coverage of extraction results to the standard words and improve the recall of the algorithm. In particular, as the number of keywords increases, the influence of word frequency decreases, and the advantage of increasing the recall of the algorithm in this paper will be more obvious.

Figure 9 describes the *F*-Measure of each algorithm when extracting different numbers of keywords. When evaluating the experimental results, we hope that the higher the *P* and *R* values, the better. But in fact, in most cases, the two are contradictory, so *F*-Measure should be used to comprehensively consider the two indicators. The *F*-Measure can reflect the effectiveness of the entire algorithm. For the *F*-Measure of the extraction results of the algorithms in the figure, there are the following results analysis.

1. T8 in the figure is the Word2Vec word vector clustering method, and its extraction effect alone is not good, which is consistent with the conclusion in the document [40]. It is mentioned in the document [40] that when the Word2Vec word vector clustering method is directly applied to a single document, it is not very accurate to select the clustering center as the keywords of the text, and the N words which are closest to it are not necessarily keywords. Therefore, the extraction effect obtained by using this method is general, but this method is often used in combination with other keyword extraction algorithms.
2. The T6 and T7 methods incorporate information such as the position of words into the TextRank algorithm to improve the accuracy of extraction, but the effect is worse than the T5 method because the T6 and T7 methods ignore the influence of external knowledge on keyword extraction. The comparison between T5 and T6 and T7 shows that the improved algorithm that introduces external knowledge through Word2Vec can better improve the keyword extraction effect, which is more advantageous than using a single model or feature or clustering.
3. Comparing the T5 method with the T3 and T4 methods, it is found that the three methods are the fusion of the Word2Vec model and the TextRank model. The difference is that T5 adds the statistical characteristics of words to the algorithm on the basis of considering the influence of external knowledge, which improves the deficiencies of only introducing word vector calculation to obtain keywords.
4. Comparing the T5 method with the RDD-WRank algorithm in this paper, it is found that the RDD-WRank algorithm has a better extraction effect. This is because this paper uses rough data-deduction theory to further improve the algorithm based on the fusion of the two models. Rough data-deduction can explore the potential associations between candidate keywords and increase the associated candidate words and scope. If the potential association is added to the iterative calculation of the weight of each candidate keyword, the extraction result will be more accurate, and the algorithm will be more effective.

At the same time, in order to prevent over-fitting of the experimental results of the improved algorithm, the experiment also compares the extraction results of each comparison algorithm based on datasets 2 and 3. In the experiment, the weight coefficient of the improved algorithm is set to *α* = 0.7, *β* = 0.3, and the parameters of the other comparison algorithms still take the optimal values in their respective references. The partial calculation results of the *P*, *R*, and *F*-Measure of each algorithm (retain two decimal places) are shown in Tables 2 and 3.

And, the line chart results of *P*, *R*, and *F*-measure of each algorithm are shown in Figures 10–12.

Figures 10–12 describe the comparison results of each algorithm based on the *P*, *R* , and *F*-Measure of datasets 2 and 3. It can be seen from these figures that the RDD-WRank algorithm in this paper still has a good extraction effect on the two datasets, and its three evaluation indicators are higher than that of the other methods. But for dataset 2, the precision, recall, and *F*-Measure of each method are all lower than the results of dataset 1. This is because the keywords provided in some journal articles are newly proposed key phrases by the authors themselves, but the existing word segmentation technology cannot accurately segment these phrases, which will lead to inaccurate extraction results. This is also a direction that we can study in the future. And, it is found that when the number of keywords is greater than 8, the extraction effect of the T6 method is better. Because of the influence of the text type, when the number of extracted keywords is small, the influence of word position will not be dominant in the extraction process. However, as the number of extracted words increases, keywords in professional texts such as academic paper abstracts will frequently appear at the beginning and end of the abstract. At this time, the advantages of the T6 method based on word position distribution weighting will be more prominent, and its extraction effect will be better. For each journal article, the number of keywords provided by the author generally remains around 3–6, so after the value of the number of keywords is 6, the *F*-Measure of each comparison algorithm has a downward trend. But, compared with other comparison algorithms, the extraction effect of this algorithm based on this dataset is still better. Compared with dataset 2, the extraction results of each algorithm for dataset 3 will be better. This is due to the fact that the effective keywords proposed in reference [47] are referred to when manually labeling keywords in dataset 3. The effective keywords here refer to the information that is valuable to users and businesses in the comments, and most of such key information is common vocabulary. The existing word segmentation technology is easy to perform accurate segmentation, and the extraction effect will be more accurate.

Based on the above analysis, the precision (*P*), recall (*R*), and comprehensive evaluation index *F*-Measure of the algorithm in this paper are higher than those of the other comparison algorithms, which shows that the TextRank algorithm using word vector clustering based on rough data-deduction and fusing with the Word2Vec model is more effective in extracting results. The TF-IDF algorithm based on statistical characteristics and the other several algorithms are more dependent on the word frequency in essence, and may preferentially extract frequently occurring words. But for a document, especially Chinese text, the subject words may not always appear. Therefore, the TextRank algorithm based on rough data-deduction starts from the text as a whole, expands the scope of association, increases the associated data, and establishes the association between words through rough data-deduction, which can further improve the accuracy of the algorithm.

## 7. Conclusions

Through research on text keyword extraction, it is found that the potential association between words and external knowledge has a direct impact on keyword extraction results. Therefore, based on rough data-deduction, this paper proposes a TextRank keyword extraction algorithm combined with Word2Vec model. It can obtain more external knowledge information to use rough data-deduction to explore potential associations between candidate keywords and use word embedding technology to integrate Word2Vec into the algorithm. The experimental results show that the improved algorithm of word vector clustering based on rough data-deduction takes into account the potential associations between candidate words and external knowledge, which further improves the accuracy of keyword extraction. In the next step, we will further refine and improve the rough data-deduction rules to obtain better extraction results.

## Figures and Tables

**Figure 1:** CBOW and Skip-Gram model structures.

**Figure 2:** Diagram of rough data-deduction in keyword extraction.

**Figure 3:** The distribution of words in HowNet and Cilin.

**Figure 4:** Flow chart of improved algorithm.

**Figure 5:** The *F*-Measure of extraction results under different *α*. *α* and *β*.

**Figure 6:** The *F*-Measure of extraction results under different *ω* values.

**Figure 7:** Comparison of *P* values of various algorithms.

**Figure 8:** Comparison of *R* values of various algorithms.

**Figure 9:** Comparison of *F*-Measure of various algorithms.

**Figure 10:** *P* value of each algorithm. (a) Results based on dataset 2. (b) Results based on dataset 3.

**Figure 11:** *R* value of each algorithm. (a) Results based on dataset 2. (b) Results based on dataset 3.

**Figure 12:** *F*-Measure of each algorithm. (a) Results based on dataset 2. (b) Results based on dataset 3.

**Table 1:** Comparison of experimental results of various algorithms.

Keywords (pcs)	Algorithm	*P* (%)	*R* (%)	*F* (%)
3	T1	47.71	14.31	22.02
	T2	64.22	19.27	29.64
	T3	66.36	19.91	30.63
	T4	28.13	8.44	12.99
	T5	67.28	20.18	31.05
	T6	61.16	18.35	28.23
	T7	62.08	18.62	28.65
	T8	55.96	16.79	25.83
	RDD-WRank	69.75	20.93	32.19

4	T1	44.04	17.61	25.16
	T2	56.19	22.48	32.11
	T3	61.24	24.50	34.99
	T4	28.21	11.28	16.12
	T5	62.61	25.05	35.78
	T6	57.11	22.84	32.63
	T7	58.26	23.30	33.29
	T8	51.83	20.73	29.62
	RDD-WRank	63.43	25.37	36.24

5	T1	41.65	20.83	27.77
	T2	53.21	26.61	35.47
	T3	56.15	28.07	37.43
	T4	27.52	13.76	18.35
	T5	57.61	28.81	38.41
	T6	53.94	26.97	35.96
	T7	55.41	27.71	36.94
	T8	47.34	23.67	31.56
	RDD-WRank	59.26	29.63	39.51

6	T1	39.30	23.58	29.47
	T2	49.69	29.82	37.27
	T3	52.29	31.38	39.22
	T4	26.91	16.15	20.18
	T5	54.74	32.84	41.06
	T6	51.07	30.64	38.30
	T7	51.22	30.73	38.42
	T8	46.18	27.71	34.63
	RDD-WRank	55.86	33.52	41.90

7	T1	37.79	27.16	31.95
	T2	46.66	32.66	38.42
	T3	49.93	34.95	41.12
	T4	27.00	18.90	22.23
	T5	50.98	35.69	41.99
	T6	49.02	34.31	40.37
	T7	48.10	33.67	39.61
	T8	44.43	31.10	36.59
	RDD-WRank	54.10	37.87	44.55

8	T1	36.99	28.26	32.66
	T2	44.15	35.32	39.25
	T3	46.44	37.16	41.28
	T4	26.61	21.28	23.65
	T5	47.48	37.98	42.20
	T6	46.56	37.25	41.39
	T7	45.76	36.61	40.67
	T8	43.35	34.68	38.53
	RDD-WRank	50.93	40.74	45.27

9	T1	35.12	30.31	33.12
	T2	42.00	37.80	39.79
	T3	44.34	39.91	42.01
	T4	25.99	23.39	24.63
	T5	45.16	40.64	42.78
	T6	44.14	39.72	41.82
	T7	43.63	39.27	41.33
	T8	42.41	38.17	40.17
	RDD-WRank	48.97	44.07	46.39

10	T1	32.98	32.98	32.98
	T2	39.72	39.72	39.72
	T3	42.20	42.20	42.20
	T4	25.05	25.05	25.05
	T5	42.66	42.66	42.66
	T6	42.57	42.57	42.57
	T7	41.83	41.83	41.83
	T8	41.19	41.19	41.19
	RDD-WRank	47.27	47.27	47.27

**Table 2:** Comparison of experimental results based on datasets 2 (Top*N* takes 3, 5, 7, 10).

Keywords (pcs)	Algorithm	*P* (%)	*R* (%)	*F* (%)
3	T1	16.03	11.39	13.30
	T2	9.79	6.82	8.03
	T3	7.61	5.32	6.25
	T4	6.39	4.51	5.29
	T5	15.42	10.86	12.73
	T6	15.42	10.89	12.75
	T7	16.10	11.35	13.29
	T8	16.41	11.57	13.56
	RDD-WRank	16.44	11.67	13.63

5	T1	12.90	15.28	13.97
	T2	7.96	9.27	8.55
	T3	6.53	7.62	7.02
	T4	5.96	6.99	6.43
	T5	12.76	15.01	13.78
	T6	13.57	16.02	14.68
	T7	13.46	15.82	14.53
	T8	13.06	15.33	14.09
	RDD-WRank	14.41	17.06	15.60

7	T1	11.06	18.31	13.77
	T2	6.88	11.24	8.53
	T3	5.51	9.02	6.83
	T4	5.74	9.46	7.14
	T5	10.60	17.45	13.17
	T6	11.78	19.49	14.66
	T7	11.19	18.43	13.91
	T8	10.90	17.95	13.55
	RDD-WRank	12.32	20.43	15.35

10	T1	8.89	20.99	12.47
	T2	5.68	13.24	7.94
	T3	4.70	10.98	6.57
	T4	4.82	11.32	6.75
	T5	8.22	19.35	11.53
	T6	10.36	24.55	14.55
	T7	8.38	19.71	11.75
	T8	8.49	19.98	11.90
	RDD-WRank	9.75	23.09	13.69

**Table 3:** Comparison of experimental results based on datasets 3 (Top*N* takes 3, 5, 7, 10).

Keywords (pcs)	Algorithm	*P* (%)	*R* (%)	*F* (%)
3	T1	38.39	13.82	20.33
	T2	44.38	15.98	23.50
	T3	51.87	18.68	27.47
	T4	5.24	1.89	2.78
	T5	57.87	20.84	30.64
	T6	52.81	19.02	27.96
	T7	47.19	16.99	24.99
	T8	31.84	11.46	16.86
	RDD-WRank	57.87	20.84	30.64

5	T1	39.44	23.67	29.58
	T2	42.25	25.35	31.69
	T3	49.55	29.73	37.17
	T4	5.73	3.44	4.30
	T5	51.69	31.02	38.77
	T6	47.30	28.39	35.48
	T7	43.37	26.03	32.53
	T8	35.62	21.38	26.72
	RDD-WRank	52.47	31.49	39.36

7	T1	40.29	33.85	36.79
	T2	41.01	34.46	37.45
	T3	44.38	37.29	40.53
	T4	6.50	5.46	5.94
	T5	46.71	39.24	42.65
	T6	43.02	36.14	39.28
	T7	42.46	35.67	38.77
	T8	38.44	32.30	35.10
	RDD-WRank	47.75	40.12	43.61

10	T1	37.42	44.91	40.82
	T2	37.70	45.25	41.13
	T3	37.58	45.11	41.01
	T4	6.91	8.29	7.54
	T5	39.04	46.86	42.60
	T6	38.20	45.85	41.68
	T7	37.98	45.58	41.43
	T8	36.24	43.49	39.53
	RDD-WRank	42.02	50.44	45.85

## Data Availability

The data used to support the findings of this study are included within the article.
